# Health Index Estimation of Wind Power Plant Using Neurofuzzy Modeling

**DOI:** 10.1155/2022/9535254

**Published:** 2022-05-29

**Authors:** Shahanaz Ayub, Rajasekhar Boddu, Harshali Verma, Sri Revathi B, Bal Krishna Saraswat, Anandakumar Haldorai

**Affiliations:** ^1^Electronics and Communication Engineering Department, Bundelkhand Institute of Engineering and Technology, Uttar Pradesh, Pin-284128, Jhansi, India; ^2^Department of Software Engineering, College of Computing and Informatics, Haramaya University, Dire Dawa, Ethiopia; ^3^Digital Communication, Bundelkhand Institute of Engineering and Technology, UP, Jhansi, India; ^4^School of Electrical Engineering, Vellore Institute of Technology, Chennai, India; ^5^Department of Computer Science & Engineering, Faculty of Engineering & Technology, SRM Institute of Science & Technology, NCR Campus, Modinagar, 201204, Ghaziabad, Uttar Pradesh, India; ^6^Department of Computer Science and Engineering, Sri Eshwar College of Engineering, 641202, Coimbatore, Tamil Nadu, India

## Abstract

According to the Tamil Nadu Energy Development Agency (TEDA) in the 2019-20 academic year, the wind power plant produces 23% of the biomass power supply in the Indian electrical commodities. To maintain the power withstanding capability needed for future electrical commodities, a yearly power shutdown program is implemented. An additional wind power plant unit will be erected and create more electricity, thereby balancing India's commercial electricity needs. Even in a nonstationary working environment, continuous monitoring and analyzing the efficiency of wind turbines is a more difficult task. Consequently, in this paper, a health index calculation for wind power plants is proposed utilizing neurofuzzy (NF) modeling. Wind generator efficiency can be measured mathematically by recording three crucial primitivistic such as observed rotation speed, generation wound temperature, and gearbox heat. Fuzzy rules are used to design the parameters of the neural network (NN), and the accumulated signal is compared using the nonlinear extrapolation approach to determine the wind generator's behavior and evaluate the hazards. During the experimental study, two windows of 24 hours and 60 hours are used, where the deviation signal required for the hazard induction is investigated. The proposed approach can accurately calculate the wind generator's health state. As a result of an improved health operating and management (HOM) system, the amount of power generated by industrials and domestic appliances has increased dramatically.

## 1. Introduction

Wind turbines have a lower fuel cost than other renewable energy sources in large-scale applications [1–3]. A wind generator's efficacy might fluctuate depending on the situation due to various geological characteristics, climate conditions, and wind farm characteristics [4, 5]. Power suppliers will have more useful data to aid in power generation planning if the total output of windy power plants (WPP) can be projected with high precision [6]. With this information, a WPP may be managed in a flexible and intelligent way (e.g., enhanced wind farm operating schedules and reactive energy flow). Estimating wind power generation can be done using physical procedures, analytical methodologies, fuzzy-based techniques [7], and even hybrid approaches [8]. Because of the detection and tracking limitations imposed by WPP's detectors and tracking systems, physical techniques must rely mostly on numerical weather forecasts [9]. Variable factors, calculation time, time limitations, and sampling frequency all affect WPP's capacity to provide reliable information. It is easier to predict the efficiency of a single wind turbine than the entire WPP's output [10]. Low-cost forecasting methods based on probabilistic and neuronetworking principles are available. A nonlinear model of the interactions between input and output information can be created based on previously observed information. However, the anticipated error may be large if additional data that was not previously included in the collection of retraining data is used as intake into such a type of system [11].

According to [11], wind farms have a large prediction error and a wide range of failures. If an abnormal wind farm is not discovered and corrected in a timely manner, it could cause lengthy outages and even lead to a lack of electricity generation. Wind farms, on the other hand, have a major challenge due to their high operational expenses. Because of this, it is becoming increasingly important to improve wind turbine O&M technology such as state tracking and wind farm problem diagnostics [12]. Evaluating wind turbines' real-time operational conditions and discovering emergent faults requires conducting an electronic health review. Administrators of wind farms can use it as a timely reminder to prioritize and construct time-based condition-based repair plans. A wind farm's operating costs and loss risk can be reduced by monitoring the operational state of all its wind generators [13]. Consequently, the safety and efficiency of the wind farm have been improved.

There is still a lot of work to be done in terms of healthcare performance measurements and assessment concepts, which are still in the early phases of development [14]. The three types of wind farm healthcare evaluation strategies outlined in the research include neural network- (NN-) based approaches, knowledge-based techniques, and data-based techniques [15]. Many various components and functions make up the wind farm's electromechanical structure. In addition, the many elements' linkages are intricate. It is so difficult to construct a precise numerical model for a wind farm of this size and complexity [16].

Assessment of wind turbine maintenance will raise several difficulties, the majority of which are addressed in the following sections. To begin, the wind farm will receive numerous (false) alerts due to multiple state tracking systems and the segregation of designs in subassemblies of the wind farm (separate modeling for gearboxes, one modeling for bearings, etc.) [17]. As a result, it is nearly impossible to keep track of operations. Furthermore, because there is only one model for each WT, wind farms with many large wind farms will be impossible to operate. As a result, it is difficult to scale state monitoring equipment in large wind farmlands. Keeping track of each WT's data for a long period of time would be the next challenge in setting alarm thresholds. Because of the lack of standardization in the system's characteristics, operations are more costly as a result. Consequently, it is necessary to significantly improve the status tracking methods [18].

A lot of attention is being paid to NN-based systems (especially multilayered perceptron), which can handle nonlinear effects. When developing a neural network model, it is customary to use characteristics such as GWT, rotation speed (RS), windy speed (WS), gearbox temperatures (GT), AT, and pitching angle PA, as well as NT, to anticipate the resultant active energy (AP) for such WT. Anomalies are recognized in the same way as in anomaly identification methods when the gap between expected and observed AP is greater than a specified level [19]. Several of the new components of the study mentioned in this research are the utilization of this signaling to construct a probabilistic health state model for such a WT because it has data about its healthcare.

In this paper, a health index calculation for wind power plants is proposed. Wind generator efficiency can be measured mathematically by recording three crucial primitivistic such as rotation speed, generation wound temperature, and gearbox heat. Fuzzy rules are used to design the parameters of the neural network (NN). The proposed approach can accurately calculate the wind generator's health state. During the experimental study, two windows of 24 hours and 60 hours are used, where the deviation signal required for the hazard induction is investigated.

The rest of the paper is structured as follows: Section 2 focuses on related work, in which the authors' contributions to wind power plant healthcare are examined. A neurofuzzy model and mathematical approach to changing window sliding are discussed in Section 3. For operating and management systems, Section 4 presents experimental findings that demonstrate how well the wind generator's healthcare parameters are evaluated. Finally, Section 5 provides a conclusion and a look at what the future holds.

## 2. Literature Review

For the most part, condition monitoring systems (CMS) in this industry demand a deeper knowledge of the monitored process. Sadly, this information is hard to obtain by and often does not exist [20]. Physical representations of such a network are rarely generated with great precision because of its complex interplay across several dynamical components. Furthermore, vibrations are the primary focus of the current CMS. As a means of assessing the health of machines, vibration testing has recently gained in popularity [21]. Unfortunately, vibrating detectors are rarely installed on all rotors and modules due to their high cost. A lack of state tracking has resulted in many turbines that are merely equipped with a vibrating sensor at each of their primary components. On the other hand, it appears that a large amount of operational (SCADA) data will be used to determine the generator's status. According to [22], wind farm CMS construction is the most cost-effective when such data is used. Data on the state of the turbine or observations of indicators such as current flow, temperatures, or tensions will be used as performance information in the turbine.

Using turbine condition data, problems can be predicted 5–60 minutes in advance in [23]. Performing preventive maintenance during this predicted timeframe would be difficult due to the lack of time available for workers to complete tasks. Signal processing techniques that focus on the trending of key data or combinations of signals can be used to detect major fluctuations in turbine performance at an early stage. Using neural network (NN) design techniques, [24] shows that signaling activity can be predicted weeks, days, and even months in advance. These methods are more suited to allowing workers to correct problems before the component fails [25]. Model-based techniques are used to build conventional behavioral patterns that can predict a specific output signal when given one or more data inputs [25]. Many signals could be discovered to be linked to other information monitored simultaneously, such as wind speed or power generation. This is perfect for wind farm signaling. To analyze wind farm signals, the use of a typical behavioral notion is advantageous because it does not require any prior knowledge of signaling behavior. The availability of signal tracking seems to be a fundamental component of the normal behavioral idea, as mentioned, as well [26].

When the turbine parts are considered normal (usually functional), which is typically at the beginning of the device's lifespan, the conventional behavioral modeling is constructed. Learned systems are then used to predict signals, and the forecasting error indicates signal behavioral changes that lead to flaws in the system. The scientific community is quite interested in this technique [26]. Autoregressive using exogenous input (ARX) modeling is used in this case to determine the status of a wind farm generator bearing using SCADA signals. Unfortunately, this approach involves human involvement in variable selection to produce a decently functioning system. Due to the large number of signals and generators that need to be inspected, human activity must be restricted. It is common for many operations to apply artificial intelligence approaches (learning capacity), and SIMAP and MARS are two of the most recent sophisticated technology that employs this strategy (MAS). There are two ways to create SCADA information typical behavioral models using artificial neural networks [27]. Such a NN design approach is often pursued, with the creation and demonstration of NN's exceptional efficiency in this scenario being one of the most common examples. Wind farm drive train parts were tracked using neural networks (NNs) in prior investigations in [28].

In [29], it is suggested that additional research be conducted on the impacts of duration, deterioration, and failure predicting, as well as anomaly identification on the state tracking of such a specific section of WT (generating heat). In addition, regression techniques are used to develop a polynomial framework for predicting the generation of heat. The system's input variables are generated output and additional variables created by integrating generator ambient temperatures (AT), nacelle temperatures (NT), and coolant temperature. By using its descriptive language, the system is used to improve total power generation while also providing an empirical basis for managing a single subassembly. A later version of the system will incorporate enhancements to allow its use in real-world WT scenarios that may include varying environmental conditions. While considering the ninth-degree polynomials, the energy curve of a WT is often the primary focus of research publications in this area that use descriptive modeling. However, most of the descriptive modeling for WTs are in research centers upon endurance, fault detection, and deterioration of the devices. As a result of the failure of the dataset or simulations, proportionate hazard modeling (PHM) was employed in this scenario. Diagnostics rely heavily on the usage of PHMs, a sort of failure model [30]. Covariates and a baseline are the two main components of this typical design.

## 3. System Model

To evaluate a WT's current and comprehensive health status, the healthcare state tracking alerts if the established health state signal deviates from expected regular healthcare circumstances. As a result, the system's application can be characterized as precautionary actions necessary to ensure a successful performance. Such a paper suggests a method for developing a parameterized health situation surveillance design (like a usual behavioral concept) that monitors the WT's actual time as well as actual health situation via its subassemblies but also elevates an aware flag when such WT's ailment deviates from the anticipated normal situation. To achieve that, NN modeling will be first built for every characteristic under consideration (GT, RS, and GWT). The deviating signal is then recovered, and that is responsive to variations in the healthy state of every characteristic. Next, using these signals, a parameterization model with such a PHM-based shape for every one of the characteristics is created. Depending upon the effectiveness of such NN and PHM-based modeling, such produced designs having PHM aspects are integrated to generate the ultimate incremental parameterized health state modeling of such WT. This final design is utilized to evaluate the WT's entire condition in actual time, providing support to the controller and assets administration group in improving performance and servicing schedule.

The HMS created in this study seeks to recognize features and structures in SCADA information, in addition, to anticipating potential problems, allowing wind farm operators sufficient time to adjust servicing schedules or undertake other precautions to avoid unplanned hardware failure. For it though, 10 minutes averaging SCADA information that are routinely accessible to controllers are employed.  Figure 1 depicts the basic structure of such HMS that was created. The functions of the various HMS units (see Figure 1) are discussed here.

### 3.1. Training Module

When modeling is still not accessible or further learning is necessary, the typical behavior modeling is learned within the learning program. If an element is changed as well as the signaling relationships alter as a result, the converse is accurate. The dataset is normalized before building the models using the methods provided, which comprises a validation checking, a dataset ranging check, and absent data analysis, as well as latency elimination. Various training stages are provided in the learning program to enable quick evaluation. Over one month of continuous practical data collecting, the initial model development is undertaken. If three, six, and following nine months additional information is collected, more workouts are conducted. The developed ANFIS system and standardized criteria designating the typical operating region of wind generators utilizing the estimation inaccuracy are the outputs of such a learning program.

### 3.2. Prediction Module

When one training modeling of the sampled signal is accessible on a modeling basis, the forecasting unit becomes operational. The predicted inaccuracy is computed and saved using the created normal behavioral framework.

### 3.3. Anomaly Recognition Module

Discrepancies in forecast mistakes are found in this section. This will be done using the learning module's calculated normal behavior criteria but rather expert-defined parameters. The result is an anomalous matrix with data on the incidence but also the date of incidence and the present anomaly's period on weekdays.

### 3.4. Initializing Module for Fuzzy Experts

Number of intakes and outlets, and also respective MFs, are initialized as in FIS frameworks utilized for anomaly detection and element conditional assertions. Every element that needs to be checked will have its unique FIS, whereas the inputs vary depending on the element or system being investigated, and every FIS architecture includes the corresponding output data: diagnostic (details regarding the signal's aberrant activity) state possible root causes.

### 3.5. Fuzzy Expert Application Module

Using the forecasting failures and data about current abnormalities, the updated FIS architecture is assessed within that component. The result is saved in a textual form then displayed to provide the analyzer with a complete picture of such turbine's state.

NN has been made up of neurons, whose parameters are interpolated among the input parameters as well as the targeted variable via an optimizing process (e.g., gradient of weighted conjugates). For ordinary behavioral analysis of GT, GWT, and RS impulses, a multilayered perceptron feed-forward neural network will be used in this paper. Among the inlet and outlet nodes, it has a unique architecture wherein one or more buried tiers with various counts of neurons occur. Furthermore, the architecture lacks interaction between tiers and neurons, allowing data to pass simply from the source to the destination tier.

(1) $$\begin{array}{c} V=\left\{v_{1},v_{2},\cdots ,v_{n}\right\},\\ {\text{AF}}_{1}=f_{1}\left(w_{i}^{h}v_{i}^{\text{in}}+b^{h}\right),\\ {\text{AF}}_{2}=f_{2}\left(w_{i}^{o}v_{i}^{h}+b^{o}\right). \end{array}$$

Every layer's result gets computed using the *V* transferring functional (or activating function) as well as input variables. Biased variables in the export layer, bias variables in the buried layer, activating functional of the buried layer, and activating functions of the exit layer are represented by *b*^*o*^, *b*^*h*^, and *AF*_1_ as well as *AF*_2_, correspondingly. Because this research has two levels, two transferring equations are used. The first transferring functional (*f*_1_) predicts the buried layer's results as well as is specified like a sigmoid functional of hyperbolic tangential pattern, as shown below.

(2) $$\begin{array}{c} f_{1}\left(w_{i}^{h}v_{i}^{\text{in}}+b^{h}\right)=\frac{2}{1+e^{-2\left(w_{i}^{h}v_{i}^{\text{in}}+b^{h}\right)}}-1. \end{array}$$

Transferring functional 2 (*f*_2_) determines the exit layer's result and is described as a sequential transferring function, as shown below.

(3) $$\begin{array}{c} f_{2}\left(w_{i}^{o}v_{i}^{h}+b^{o}\right)=w_{i}^{o}v_{i}^{h}+b^{o}. \end{array}$$

The performing metric, that is employed in learning, seems to be the summation of squared erroneous (SSE). A guided training approach called scaling conjugated gradients is used to build the NN. This approach analyses the incoming dataset then adjusts its NN's values and impairments to reduce SSE.

(4) $$\begin{array}{c} \text{SSE}=\overset{n}{\underset{j=1}{\sum }}{\left(O_{j}-O_{j}^{`}\right)}^{2}, \end{array}$$

in which *O*_*j*_ is the predicted value while *O*_*j*_^`^ is the result of NN across *n* incoming data sets. The NNs' correctness is determined using a linear extrapolation among the NN result as well as the destination parameters, with the highest attainable efficiency of 100%.

#### 3.5.1. Preprocessing

The information set utilized in the suggested approach comes from such a WT that did not have any notable failures or anomalies over one year. Erroneous data sets must be cleaned out to format such data for examination. Four filters are being created and implemented for such an objective. Filter tries to replace not-a-number (NaN) results with such an averaging value created as from NaN point's following and preceding accessible data sources. Every WT variable has such a realistic and established limit, while data sets outside of such limits are filtered out. (e.g., AP was found to be negative). It is worth noting that such filters are however implemented to produce clear information for the systems in mind. Moreover, because the WT behaved normally, the results cannot go beyond a confidence level. For example, to be labeled unusual, two of three successive data values have to be beyond a set range. Filter incorporates this under account using power-curve measurements, while filter adjusts and adjusts every variable in a defined limit now at a conclusion.

The sources are however verified to ensure that such recorded values for every parameter approximate the dispersion of such optimum values. It stops the system from producing an output based on uncertain input data, which helps to reduce the model's inaccuracy. Modeling for characteristics using NN, these NN types are created in this stage to imitate the typical functioning of GWT and GT, as well as RS. This NN for such three NN types seems to be a multilayered perceptron feed-forward having the architecture of one concealed layer having 50 neurons and also one convolution layer. The AP, NT, and AP-1, as well as AP-2 along with the matching GT as well as GWT predictor parameter, represent the inputs to NNGT as well as NNGWT. AP-1, as well as AP-2, is still the A*P* values obtained from the two preceding periods. The purpose of including such two factors is to look at the effect of the previous action on ongoing operations. The WS, as well as AP, seems to be the NNRS's sources, having RS as the objective parameter. A year's worth of information (37,000 measuring values) averaging at 10-minute intervals was arbitrarily split into 70 percent, 15%, and 15% for learning, testing, and verification, correspondingly.

The “randomized” sample method was selected since it ensures that every collected data is similarly likely, such that 70 observations are picked for learning, 15 for tests, as well as 15 for verification out of each 100 observations. Even though it may lessen some relationships among some associated activity moments in duration, it has proven to become the most effective method. When “block-type” but rather “time-dependent” sample strategies are used, for example, they directly split specific intervals and limit the system from learning as many potential structures as feasible, which constitutes a disadvantage. The studies are being conducted to prevent several of the challenges that come with interacting using NNs, like overfitting.

As a result, the system is only allowed after every testing, whereas if changes in efficiency among the “learning,” “testing,” and “verification” data points are lower than 0.1 percent. As a result, just one graph reflects the entire dataset, like all three charts (learning, tests, and verification) are identical with 0.1 percent error, as shown in Figure 2. Instead, the modeling will be modified since this requirement is satisfied. Similarly, this knowledge is gained through running numerous tests and examining the model's results. After applying this requirement, the aggregate defect rates for every NN system are calculated by averaging the prediction error from the three databases. Furthermore, when a subassembly gets removed or the element is significantly modified, a separate NN system must be developed.

For highlighting and explaining the suggested parameterized model's characteristics, the established parameterized health state concept will be of relevance in a variety of ways, including how it handles many of the existing issues identified in such a current research review. It must be noted that such a paper proposes a way for modeling health conditions, and the generated model's parameterized shape will be a big characteristic. Furthermore, all studies are conducted by observing normal performance, which can mitigate against the absence of failing facts in the environment. The system excels in the below aspects, which can be investigated deeper in subsequent research:

#### 3.5.2. Adaptability

Because most of the modeling deployed thus yet are dependent upon NNs, there seems to be a difficulty with adaptation, as NN-based estimates of specific WTs will not be used alternately. A modeling approach, on the other hand, has the benefit of being able to change the variables and reuse the prototype for different WT. In addition, to verify the improved variables, more research will be required.

#### 3.5.3. Scalability

Developing unique NN modeling for every WT in such a wind turbine having a huge minority of WTs, in which the commonalities among simulations will not be simply studied, is a challenge for the field administrator and controller. One such research can be carried out using the suggested concept, and contrasts of simulations among a low minority of WTs will lead to a generic concept for such farmland. Evaluation of the residual usable lifetime is as follows: the parameterized approach presented herein will be for a one-year study span in which the WT does not experience any significant anomalies. This means the actual behavioral and modeling will be utilized like a guide. The effectiveness of every year can then be contrasted to such figures. An alternative perspective, a comparable simulation for every year, will be built, with correlations between the variables of the simulations potentially yielding insights on the deterioration matter. Certainly, it can lead to improvements in operational planning.

## 4. Results and Discussion

Neuronetworking simulators can be used in the proposed model to test the wind generator's proposed modeling for healthcare purposes. The suggested health monitoring systems make advantage of all available fuel efficiency parameters. Certain health markers change because of the aberrant operation of the wind farm generating systems. There was a 72-hour period in which wind speed and energy data from the wind farm SCADA were compared and evaluated using three state wellness indicators based on data linkages. The results of such investigations are depicted in Figures 3 and 4. The three wellness indices changed drastically after 40 hours, indicating that the status of these wind farm generator systems was unique.

A standardized dataset correlation model was developed based on SCADA information acquired during the ordinary operation of a wind farm on its first day of operation. The following is the relationship between wind velocity and energy data, as demonstrated using wind velocity and energy statistics as an example:

(5) $$\begin{array}{c} P_{\text{std}}\left(v\right)=5316.85-2618.04v+403.17v^{2}-17.34v^{3}. \end{array}$$

The changing regulation of wind farm generator operational health indicator is generated by setting the window wide to 24 hours as well as the window increments to 1 hour.

The changing regulation of the operational health indicator of a wind farm generator is generated by setting the window width to 24 hours, and the window increments to one hour.  Figure 5 displays a graphical representation of the cumulative development of health state following administration of the *F*. Various confidence range degrees are investigated for such *Y*, and the 99 percent confidence gap produced the best results in terms of accurately matching the genuine fluctuations as well as the input information. It should be noted that such a case study based on the proposed HCWT concept was generated with information that was free of significant anomalies, which should be noted.

## 5. Conclusions

This paper that is proposed a neurofuzzy modeling to check the dynamic health state of the wind turbines through typical behavioral characteristic is obtained from discrepancy real-time signal of the wind generator. The neural network can be utilized for state tracking and anomaly identification, an incremental approach built inside healthcare state modeling which recognizes state changes as in WT's action. The proposed system seems to have a simple design having a minimal set of variables, as well as it has been validated by evaluating real and synthetic information. Fuzzy logic can naturally handle available expertise information regarding anomaly/prediction mistake pattern analysis and underlying causes identification. Once criteria are specified, automatic fault diagnosis becomes possible. Hence, the accuracy rate, is contingent on the availability of varied SCADA signals, is addressed. Such requirement is frequently met, allowing the proposed system is applied to both current and newer rotors. Therefore, it has identified current problems in SCADA data and gives broad status and diagnosis remarks. Furthermore, the proposed model is implemented in the authorized private wind power plant to study practical circumstance facing by the wind generator.

## Figures and Tables

**Figure 1:** The proposed health management systems (HMS).

**Figure 2:** Structure of multilayer neural networks.

**Figure 3:** Performance of the health indicator of the wind turbine.

**Figure 4:** Performance of the power degradation indicator of the wind turbine.

**Figure 5:** Cumulative health condition indicator of the wind turbine.

## Data Availability

The data used to support the findings of this study are available from the corresponding author upon request.

## References

[1] International Energy Agency (2019). Offshore wind outlook 2019. *World Energy Outlook Special Report*.

[2] International Renewable Energy Agency (2019). Future of Wind: Deployment, Investment, Technology. *Grid Integration and Socio-Economic Aspects*.

[3] Freeman K., Frost C., Hundleby G. (2019). Our energy, our future. *How offshore wind will help Europe go carbon-neutral*.

[4] Song Z., Zhang Z., Jiang Y., Zhu J. (2018). Wind turbine health state monitoring based on a Bayesian data-driven approach. *Renewable Energy*.

[5] An X., Zeng H., Yang W., An X. (2017). Fault diagnosis of a wind turbine rolling bearing using adaptive local iterative filtering and singular value decomposition. *Transactions of the Institute of Measurement and Control*.

[6] Yang W., Liu C., Jiang D. (2018). An unsupervised spatiotemporal graphical modeling approach for wind turbine condition monitoring. *Renewable Energy*.

[7] Deveci M., Cali U., Kucuksari S., Erdogan N. (2020). Interval type-2 fuzzy sets based multi-criteria decision-making model for offshore wind farm development in Ireland. *Energy*.

[8] Abdel-Basset M., Gamal A., Chakrabortty R., Ryan M. (2021). A new hybrid multi-criteria decision-making approach for location selection of sustainable offshore wind energy stations: a case study. *Journal of Cleaner Production*.

[9] Niemann H., Kjølstad Poulsen N., Mirzaei M., Henriksen L. C. (2018). Fault diagnosis and condition monitoring of wind turbines. *International Journal of Adaptive Control and Signal Processing*.

[10] De Azevedo H. D. M., Araujo A. M., Bouchonneau N. (2016). A review of wind turbine bearing condition monitoring: state of the art and challenges. *Renewable and Sustainable Energy Reviews*.

[11] Liu Q., Sun Y., Wu M. (2021). Decision-making methodologies in offshore wind power investments: a review. *Journal of Cleaner Production*.

[12] Argin M., Yerci V., Erdogan N., Kucuksari S., Cali U. (2019). Exploring the offshore wind energy potential of Turkey based on multi-criteria site selection. *Energy Strategy Reviews*.

[13] Deveci M., Ozcan E., John R., Pamucar D., Karaman H. (2021). Offshore wind farm site selection using interval rough numbers based best- worst method and MARCOS. *Applied Soft Computing*.

[14] Deveci M., Ozcan E., John R., Covrig C.-F., Pamucar D. (2020). A study on offshore wind farm siting criteria using a novel interval-valued fuzzy-rough based Delphi method. *Journal of Environmental Management*.

[15] Ullah K. (2021). Picture fuzzy Maclaurin symmetric mean operators and their applications in solving multiattribute decision-making problems. *Mathematical Problems in Engineering*.

[16] Martinez A., Iglesias G. (2021). Multi-parameter analysis and mapping of the levelised cost of energy from floating offshore wind in the Mediterranean Sea. *Energy Conversion and Management*.

[17] Kheirabadi C., Nagamune R. (2019). A quantitative review of wind farm control with the objective of wind farm power maximization. *Journal of Wind Engineering and Industrial Aerodynamics*.

[18] Randall R. B. (2011). *Vibration-Based Condition Monitoring*.

[19] Yang W., Jiang J. Wind turbine condition monitoring and reliability analysis by SCADA information.

[20] Kusiak L., Li W. (2011). The prediction and diagnosis of wind turbine faults. *Renewable Energy*.

[21] Schlechtingen M., Santos I. F. (2011). Comparative analysis of neural network and regression based condition monitoring approaches for wind turbine fault detection. *Mechanical Systems and Signal Processing*.

[22] Süttmann M. (2010). Master thesis: condition monitoring in wind turbines – a drive train monitoring System.

[23] Abdusamad K. B., Gao D. W., Muljadi E. A condition monitoring system for wind turbine generator temperature by applying multiple linear regression model.

[24] Gebraad P. M., Teeuwisse F. W., van Wingerden J. W. A data-driven model for wind plant power optimization by yaw control.

[25] Gebraad P. M. O., Teeuwisse F. W., van Wingerden J. W. (2016). Wind plant power optimization through yaw control using a parametric model for wake effects—a CFD simulation study. *Wind Energy*.

[26] Carlini E. M., Ianniciello A., Pisani C., Vaccaro A., Villacci D. An optimised methodology to predict the wind farms production.

[27] Louie H., Sloughter J. M., Louie H., Sloughter J. M. (2014). Probabilistic modeling and statistical characteristics of aggregate wind power. *Large Scale Renewable Power Generation*.

[28] Lydia M., Kumar S. S., Selvakumar A. I. (2011). Condition based maintenance optimization for multi-component systems using proportional hazards model. *Reliability Engineering & System Safety*.

[29] Moghaddass R., Rudin C. (2015). The latent state hazard model, with application to wind turbine reliability. *The Annals of Applied Statistics*.

[30] Leturiondo U., Salgado O., Galar D., Kumar U., Ahmadi A., Verma A. (2015). Estimation of the reliability of rolling element bearings using a synthetic failure rate. *Current Trends in Reliability, Availability, Maintain Ability and Safety*.

